This article has been retracted.

# Prevention of Venous Thrombosis of Lower Limbs after Cesarean Section Based on Smart Medical Air Pressure Therapy Instrument

**DOI:** 10.1155/2022/1451881

**Published:** 2022-07-30

**Authors:** Yuanyuan Yin, Xiang Xiao, Lingyun Peng

**Affiliations:** ^1^Obstetrical Department, The Central Hospital of Wuhan, Tongji Medical College Huazhong University of Science and Technology, Wuhan, 430000 Hubei, China; ^2^Chongqing Medical and Pharmaceutical College, 401331 Chongqing, China

## Abstract

Affected by the environment, the incidence of lower extremity venous thrombosis after cesarean section is gradually increasing, and postoperative nursing is becoming more and more important. The intelligent medical air pressure therapy instrument is a common and effective postpartum nursing method. This paper studies the role of pneumatic therapeutic apparatus in the prevention of lower extremity venous thrombosis after cesarean section in smart medicine, describes its importance in nursing, and analyzes the role of pneumatic therapeutic apparatus and smart medicine combined with the postoperative nursing situation of patients with cesarean section in our hospital. In this paper, we aggregate the description text of six levels of hospital intelligent service grading evaluation. In order to show the characteristics of each level and the requirements of each level of hospital intelligent service, we can roughly see the differences between different levels. Research shows that with the construction of medical information platform, more and more medical processes rely on hospital information system, which promotes the integration of medical platform and the interconnection of medical equipment, provides convenient services for patients, and provides patients with easier access to services. At the same time, the massive data generated by appointment, nursing, treatment, and other activities will be recorded, and the pneumatic therapeutic instrument can avoid the occurrence of 60% lower extremity venous thrombosis. The data of air pressure therapeutic instrument is dynamic, and its performance is mainly reflected in the recording of dynamic index data.

## 1. Introduction

As the basis of the construction of smart hospital, the air pressure therapeutic instrument has become an important part of hospital information resources. The use and development of air pressure therapeutic instrument will become a trend. Pneumatic therapy device can cause venous thrombosis of lower extremities after cesarean section. But at present, the air pressure therapeutic instrument is still in the construction stage, and the analysis of drug use benefit and drug treatment scheme by using the method of nursing after cesarean section can provide reference for clinical medication decision-making.

Johnson et al.'s study showed that compared with simple anticoagulation, CDT has the advantages of rapid thrombus clearance, increased venous patency rate, and reduced the incidence of PTS; however, its bleeding complications increased by 2 times [1]. In recent years, Strongman et al. proposed that the effectiveness and safety of mechanical thrombectomy have been confirmed, especially for the removal of proximal iliofemoral deep vein thrombosis in the acute stage, which has been widely used in clinical practice [2]. Based on 20 retrospective case-control studies, Borchmann et al. compared the efficacy of Angiojet and CDT in the treatment of acute LEDVT [3]. Horwitz et al.'s study shows that the use rate of oxytocin in low-risk primipara before active period is increased [4]. However, the results of relevant studies are still controversial. Hohaus et al.'s study found that compared with early admission, delayed admission of pregnant women had shorter labor time and lower painless delivery rate. There was no significant difference in cesarean section rate, labor intervention, and vaginal delivery rate between the two groups [5]. We found that the pregnant women who were not satisfied with the vaginal delivery in the early stage of hospitalization were not satisfied with the vaginal delivery.

Kekre and Connors assessed the risk of VTE in 859 patients after cesarean section in Hong Kong. Overweight, old age, multiple pregnancy, obesity, and primary postpartum hemorrhage were common risk factors [6]. Borg et al. reported that DVT often occurs in lower extremity veins. In patients with non-Hodgkin's lymphoma complicated with DVT, the formation sites are mainly in upper extremity deep veins and jugular veins, followed by lower extremity veins. The incidence of pulmonary embolism and pulmonary embolism complicated with DVT is the lowest [7]. Gangaraju et al.'s study pointed out that VTE events often occur shortly after hand cesarean section and during disease care and chemotherapy [8]. Byun et al.'s study found that the incidence of VTE increased in patients after cesarean section and those with diabetes, poor physical fitness, high disease stage, and anemia [9]. Although VTE risk assessment can analyze the postpartum status of patients, there is a lack of intelligent medical devices for treatment.

This paper studies the role of pneumatic therapeutic apparatus in the prevention of lower extremity venous thrombosis after cesarean section in smart medicine, describes its importance in nursing, and analyzes the role of pneumatic therapeutic apparatus and smart medicine combined with the postoperative nursing situation of patients with cesarean section in our hospital. With the construction of medical information platform, more and more medical processes rely on the hospital information system, which promotes the integration of medical platform and the interconnection of medical equipment and provides convenient services for patients. At the same time, the massive data generated by appointment, nursing, treatment, and other activities will be recorded, and the pneumatic therapeutic instrument can avoid the occurrence of 60% lower extremity venous thrombosis. The data of air pressure therapeutic instrument is dynamic, and its performance is mainly reflected in the recording of dynamic index data. The main causes of lower extremity DVT are venous injury, slow blood flow, and blood hypercoagulability. Other high-risk factors include pregnancy, perinatal period, prolonged bed rest, surgical immobilization, and malignant tumors.

## 2. Intelligent Medical Treatment and Air Pressure Therapeutic Apparatus

### 2.1. Smart Healthcare

Driven by the realistic demand of economic and social development and the driving force of policy and technology, people's demands for hospital informatization level are getting higher and higher, which promotes the development of Internet plus medical health. The traditional hospital information system is difficult to meet the requirements of today's medical service level. Multiple factors such as national policy, economy, society, and technology promote the hospital to change to the direction of intelligence, marking that the construction of pneumatic therapeutic apparatus in China has entered a new stage [10]. The construction, analysis, and utilization of air pressure therapeutic apparatus play a basic supporting role in the construction and development of “smart hospital” [11]. With the development of Internet plus medical health, smart hospitals, with the core of wisdom service, wisdom diagnosis, and treatment and intelligent management, entered the period of rapid construction. As the core of medical big data, pneumatic therapeutic instrument has become the basis of the construction of “smart hospital.” The research on the analysis and utilization of pneumatic therapeutic instrument is of great significance for the construction of “smart hospital” [12]. In order to promote the analysis and utilization of air pressure therapeutic instrument, scholars have integrated the research framework of generation, analysis, and utilization of air pressure therapeutic instrument, elaborated the connotation of air pressure therapeutic instrument, analyzed the relationship between air pressure therapeutic instrument system and other medical information systems, combed the analysis and nursing process of air pressure therapeutic instrument, and summarized air pressure therapy from three aspects of computer-aided nursing, treatment recommendation, and management support application of instrument analysis [13]. Smart medical pointed out that the analysis and nursing of pneumatic therapeutic instrument is a higher level requirement of “smart hospital,” which will help the construction of high-level “smart hospital” [14].

There are still many problems in the construction process of air pressure therapeutic apparatus. This paper will analyze the challenges in the construction of air pressure therapeutic apparatus from the data level, model level, and application level; for example, the construction standards of air pressure therapeutic apparatus are not unified [15]. Air pressure therapeutic instrument is a detailed record of the diagnosis and treatment process of patients, and the data sharing of air pressure therapeutic instrument can better play its value [16]. The barometric therapeutic instrument system is gradually developed. The construction standards of barometric therapeutic instruments in various departments, hospitals, and medical service institutions are different and lack of top-level design and overall promotion and the phenomenon of digital island, which seriously hinders the data sharing of barometric therapeutic instrument across departments and institutions and limits the interconnection of barometric therapeutic instrument systems across regions [17]. The opening and sharing of pressure therapeutic apparatus will produce greater value. Data sharing and privacy protection are unavoidable problems. How to share, what level of opening, and how to protect patients' privacy need to be concerned [18]. The United States has accumulated a lot of successful experience in data sharing and established open data platforms, such as mimic database, to provide strong support for scientific research [19]. However, there is a lack of experience in the opening and sharing of air pressure therapeutic apparatus in China. In many cases, the data of air pressure therapeutic apparatus is only used for internal or scientific research and even becomes personal privilege and personal resource [20]. Even in most cases, a lot of data is still in the database, which cannot play its great value [21]. Therefore, we need to explore how to open and share the pressure therapeutic apparatus to play its value on the basis of protecting patients' privacy [22].

In recent years, the theory and method of nursing after cesarean section have developed rapidly, which makes the nursing method after cesarean section widely used in many fields and the worse the interpretability of the algorithm. Pregnant women are prone to lower extremity venous thrombosis after cesarean section due to anesthesia for cesarean section and lack of proper exercise. Although there are many researches on the nursing after cesarean section, the interpretability of nursing results is a difficult problem, which has seriously affected its application in specific fields, especially in the medical field [23]. If a decision can be explained, decision-makers can better evaluate its advantages and disadvantages and can be better adopted or improved [24]. Therefore, the interpretability of the results is also an important problem that we need to pay attention to and solve in the analysis of the pressure therapeutic apparatus by making better use of the nursing after cesarean section. The responsibility subject and relationship of nursing results application. There are great challenges in the identification of medical responsibility in the auxiliary nursing based on the clinical decision support of nursing results. How to clarify the responsibility subject and its relationship will better promote the application of nursing results after cesarean section. The current legal standards do not cover this problem, so we need to further improve and perfect the legal system to ensure the analysis and application of pneumatic therapeutic instrument.

### 2.2. Risk Assessment of VTE

Western countries have formulated guidelines based on evidence-based medicine and recommended that all pregnant women should be assessed for the risk of VTE, and low molecular weight heparin and other anticoagulant therapy and mechanical preventive measures should be given to high-risk groups, so as to reduce the risk of VTE and improve the adverse outcomes of pregnant women. However, China has not yet carried out large-scale risk assessment of VTE during pregnancy.

In addition, age, surgery, immobilization, and other comorbid diseases are also risk factors for thrombosis. The coefficient *g* of these risk *x* can be expressed as

(1) $$\begin{array}{c} X^{\left(0\right)}=\left(x^{\left(0\right)}\left(2\right),x^{\left(0\right)}\left(3\right),\cdots ,x^{\left(0\right)}\left(n+1\right)\right),\\ \text{G}=\overset{k}{\underset{i=1}{\sum }}\underset{q\in D_{i}}{\sum }{\left|q-n_{i}\right|}^{2}. \end{array}$$

The occurrence of thrombosis after hand cesarean section is affected by many factors. There are relatively few articles that simply analyze tumor-related factors and the occurrence of thrombosis after cesarean section. The model analyzes tumor-related factors and gastric cancer cesarean section by controlling other confounding factors. The relevance of postpartum thrombosis is as follows:

(2) $$\begin{array}{c} U=\left\{P_{1}\left|D,L,f_{2},Q,d,l\right.\;P_{2}\left|f_{1},\mu \right.\;P_{3}\left|N,M,I\right.\right\},\\ IR=\overset{U}{\underset{S-1}{\sum }}\overset{K}{\underset{d-1}{\sum }}f_{s},{DV}_{s},d. \end{array}$$

The incidence of thrombosis after cesarean section for gastric cancer in the model was 44.4% (60/135), which was significantly higher than the incidence of thrombosis in the lower limbs after abdominal hand cesarean section in other countries and also higher than the previous publication of this group. The incidence of thrombosis in the article *P* is as follows:

(3) $$\begin{array}{c} P_{\text{ikjl}}=\left\{\begin{array}{cc} \frac{n}{\Delta_{\text{ikjl}}}\sqrt{\overset{n}{\underset{s=1}{\sum }}{\left(x_{\text{ik}}\left(\varepsilon \right)‐x_{\text{jl}}\left(\varepsilon \right)\right)}^{2}\Delta_{\text{ikjl}}\left(\varepsilon \right),} & \Delta_{\text{ikjl}}>0,\\ 0, & \Delta_{\text{ikjl}}<0, \end{array}\right.\\ N_{1}=\left\{X_{1}\left(t‐4\;\Delta t\right),X_{1}\left(t‐3\;\Delta t\right),X_{1}\left(t‐2\;\Delta t\right),X_{1}\left(t‐\Delta t\right)\right\}. \end{array}$$

This may be because the patients we screened are mainly cancer patients. The cancer tissues can express different procoagulant proteins, such as tissue factor, cancer procoagulant, and release procoagulant particles *K*_2_:

(4) $$\begin{array}{c} K_{2}=\left\{X_{2}\left(t‐4\;\Delta t\right),X_{2}\left(t‐3\;\Delta t\right),X_{2}\left(t‐2\;\Delta t\right),X_{2}\left(t‐\Delta t\right)\right\},\text{VTE }\left(b\right)=2n\ln\left(\sigma \right)+n\ln\left(2\pi \right)+n\left\{\frac{n+tr\left(S\right)}{n-2-tr\left(S\right)}\right\},\\ W\left(\delta \right)=K\left(y\left(T-1\right),u\left(T-d-1\right)\right). \end{array}$$

In addition, tumor tissue promotes the formation of cancer-related thrombus through cell adhesion mechanism *Y*:

(5) $$\begin{array}{c} Y_{1}=\left\{Y_{1,1},Y_{1,2},Y_{1,3},Y_{1,4},Y_{1,5}\right\},\\ y_{i}=\beta \left(u_{i},v_{i}\right)+\overset{p}{\underset{j=1}{\sum }}\beta_{j}\left(u_{i},v_{i}\right)x_{ij}+\varepsilon_{j}\beta_{j}. \end{array}$$

In addition, in related studies, it was found that gastric cancer patients are more likely to develop venous thrombosis after undergoing surgical treatment. Tumor staging is closely related to the occurrence of thrombosis after cesarean section in tumor patients. A recent South Korean assessment of the incidence of perioperative thrombosis and risk factors for gastric cancer pointed out that the depth of tumor invasion is correlated with preoperative thrombosis. Laparoscopic surgery has been widely used in gastric cancer surgery. Some articles believe that laparoscopic surgery has a lower risk of thrombosis than traditional open surgery, but other studies believe that laparoscopic and open surgery methods are used after cesarean section. There is no statistical difference in the risk of thrombosis. In addition, an article in Vienna pointed out that regional lymph node metastasis is closely related to thrombosis, and the correlation is

(6) $$\begin{array}{c} Y_{2}=\left\{Y_{2,1},Y_{2,2},Y_{2,3},Y_{2,4},Y_{2,5}\right\},\\ {Y_{1}}^{\prime }=\text{avg}\left(Y_{1}\right),{Y_{2}}^{\prime }=\text{avg}\left(Y_{2}\right). \end{array}$$

In the study of tumor markers and the occurrence of thrombosis in pancreatic cancer, colon cancer, and ovarian cancer, it is pointed out that high levels of tumor markers (CEA, CA199, and CA125) increase the risk of thrombosis. When studying the risk of thrombosis in women with ovarian cancer, it was found that high levels of CA125 are a risk factor for thrombosis. The level of tumor markers is in the process of dynamic changes. The changes of tumor markers after cesarean section before and after operation are obvious. In the model, the correlation between the increase of tumor markers before and after the operation and the occurrence of thrombosis in the lower limbs after cesarean section is analyzed. CA125 after cesarean section is higher than that before operation by >5 U/mL, which is a risk factor for thrombosis of lower limbs after cesarean section.

(7) $$\begin{array}{c} \text{CEA}\left(d_{i},w_{j}\right)=P\left(d_{i}\right)P\left(w_{j}\left|d_{i}\right.\right);P\left(w_{j}\left|d_{i}\right.\right)=\overset{K}{\underset{k=1}{\sum }}P\left(w_{j}\left|z_{k}\right.\right)P\left(z_{k}\left|d_{i}\right.\right),\\ \text{CA}125\left(Ai,Aj\right)=\left[\log\left(\frac{\left|x_{A_{i}}-a_{A_{j}}\right|}{w_{A_{j}}}\right),\log\left(\frac{\left|y_{A_{i}}-y_{A_{j}}\right|}{h_{A_{j}}}\right),\log\left(\frac{w_{A_{i}}}{w_{A_{j}}}\right),\log\left(\frac{h_{A_{i}}}{h_{A_{j}}}\right)\right]. \end{array}$$

CA125 is both a tumor marker and an inflammation marker. High levels of CA125 are not only related to advanced tumors but also indicate an inflammatory response related to thrombosis. CA125 may be used as a monitoring indicator to predict the occurrence of thrombosis after cesarean section. In our findings, the univariate analysis of preoperative neoadjuvant chemotherapy is a risk factor for lower limb thrombosis after cesarean section for gastric cancer:

(8) $$\begin{array}{c} \text{C}=V\times \frac{n}{Q}+\frac{Q}{\left(D/2\right)2\times \pi },\\ {f_{R}}^{A_{i}}={w_{G}}^{A_{i}A_{j}}\cdot V. \end{array}$$

An article evaluating the risk of thrombosis in patients with esophageal and gastric cancer receiving neoadjuvant chemotherapy pointed out that neoadjuvant chemotherapy is an independent risk factor for thrombosis, and preoperative neoadjuvant chemotherapy is a risk factor for thrombosis after cesarean section. The mechanism of thrombosis caused by chemotherapy includes damage to vascular endothelial cells, resulting in an imbalance between procoagulant and anticoagulant molecules, inducing tumor endothelial cell apoptosis, activating cytokines, and increasing tissue factor activity:

(9) $$\begin{array}{c} {M_{n}}^{\prime }-H_{ys}>M_{p},\\ w_{G}=\max\left\{0,W_{G}\cdot \varepsilon \left({f_{G}}^{A_{i}},{f_{G}}^{A_{j}}\right)\right\}. \end{array}$$

In the model, neoadjuvant chemotherapy was not statistically significant in multivariate analysis. By calculating the remission rate of the thrombosis group and nonthrombosis group after neoadjuvant chemotherapy, it was found that the remission rate of the nonthrombosis group was higher. This indicates that patients whose curative effect is relieved by neoadjuvant chemotherapy have a reduced risk of thrombosis after cesarean section. Air pressure therapy instrument analysis and care can provide support for disease cost management. Use the postcesarean section nursing technology to analyze and identify the different diagnosis and treatment behavior patterns in the process of disease diagnosis and treatment, such as the use of medicines and sanitary materials, and explore the main factors that affect patient costs under different diagnosis and treatment behavior patterns, and analyze the disease costs based on patient information. Forecasting provides new ideas for disease cost management and control.

## 3. Experiment of Air Pressure Therapeutic Apparatus to Prevent Uterine Cervix Birth

### 3.1. Methods

This article studies the role of air pressure therapy instrument in the prevention of venous thrombosis of the lower extremities after cesarean section in smart medical care, describes its importance in nursing, and combines the postoperative care of cesarean section patients in our hospital. After inspection, it is determined that the revised content is consistent with the original intention of the author.

### 3.2. Design

In this paper, we aggregate the description text of six levels of hospital intelligent service grading evaluation. In order to show the characteristics of each level and the requirements of each level of hospital intelligent service, we can roughly see the differences between different levels. Level 0 mainly includes “manual” and “registration,” level 1 includes “appointment” and “information system,” level 2 includes “self-help” and “sharing,” levels 3 and 4 highlight “mobile” and “online,” level 5 mainly includes “monitoring” and “record management,” and the evolution of keywords also shows the changes of requirements at different levels. The analysis of air pressure therapeutic instrument will enable the practice and help the improvement of hospital intelligent service. Only 5 cases recommended low molecular weight heparin, the other 29 cases had no clear indication.

#### 3.2.1. Risk Factors

There were 369 cases of elective cesarean section, 162 cases of 35 years old, 76 cases of cesarean section during labor, 75 cases of premature delivery, 65 cases of forceps assisted delivery, 29 cases after IVF-ET cesarean section, 36 cases of preeclampsia, 30 cases of multiple pregnancy, and 51 cases of postpartum hemorrhage. All patients in the high-risk group used low molecular weight heparin to prevent VTE after assessing and excluding the risk of bleeding.

#### 3.2.2. Analysis of Relevant Risk Factors

Univariate analysis and multivariate analysis were used to analyze the clinical indicators and risk factors of VTE. Three patients developed DVT, 2 cases were pregnant, 1 case was after cesarean section, and the incidence rate was 1.28%. There was no pulmonary embolism in the model. In the model, bed rest in early pregnancy has also become a major risk factor of VTE in Chinese pregnant population, which is different from that in western countries. The proportion of bed rest in early pregnancy for 3 days is as high as 6.9%. Although there is no evidence to support bed rest in the treatment of threatened abortion, many doctors still choose bed rest as an important means of “fetal protection.”

#### 3.2.3. Characteristic Observation

The time and location of thrombus formation in patients with NHL and VTE were comprehensively analyzed. For pregnant women in China, affected by the traditional concept, especially women with previous abortion history, they are more nervous and anxious. They think that only lying still in the first trimester can secure the fetus. Therefore, the proportion of lying in bed and braking in the first trimester is significantly higher than that in western countries, which increases the risk of VTE. The general clinical data of the patients were observed, and the correlation between the clinical indicators and VTE events was analyzed.

## 4. Results and Discussion

### 4.1. Air Pressure Therapeutic Apparatus in Preventing Lower Extremity Venous Thrombosis after Cesarean Section

As shown in Figure 1, the data of air pressure therapeutic instrument is the comprehensive integration of other medical information system data with the patient as the center, and the representation form is diversified. The data of air pressure therapeutic instrument includes not only unstructured data such as text description of patients but also structured data such as examination and test reports. For specific patients, the pneumatic therapeutic instrument mainly includes admission records, course records (including the first course records and other course records), inspection reports, treatment records (such as operation records), and discharge summary. The air pressure therapy device stimulates acupoints, accelerates blood flow, and massages muscles to promote body metabolism and reduce the formation of lower extremity venous thrombosis. The air pressure therapeutic instrument records the important diagnosis and treatment information of patients, which has the potential to provide huge support for clinical decision-making, clinical research, and application management. Therefore, it is necessary to analyze the data of the air pressure therapeutic instrument and enable nursing practice.

As shown in Figure 2, the collection, extraction, storage, and processing capacity of medical data are growing rapidly. In the face of massive medical information, theoretical methods such as nursing after cesarean section will help the analysis and utilization of pneumatic therapeutic apparatus and provide better support for relevant decision-making. The analysis and utilization framework of air pressure therapeutic apparatus based on nursing after cesarean section are shown in Table 1.

In current clinical practice, many treatment methods are lack of effective evidence support. Although reference guidelines are used to assist decision-making, they are usually based on randomized controlled trials (RCTs). However, RCT patient cohort is limited, and standard is strict and has been carefully designed to reduce the universality. Traditional RCT research also faces many limitations, such as rare disease research and less clinical case support, and contains other factors that are difficult for patients to control. In addition, due to the limitation of ethics, some interventions are difficult to implement and RCT research cannot be carried out.

As shown in Figure 3, due to various limitations, RCT only supports part of clinical decisions, most of which have no evidence to follow. The data of air pressure therapeutic instrument is the data archiving record in the process of diagnosis and treatment of patients, which contains a lot of information and knowledge and has the value of analysis, utilization, and further nursing. Compared with RCT and prospective cohort studies, the use of pneumatic therapy can greatly reduce the cost of research and can also implement the research that cannot be carried out before, reduce the difficulty of research, and provide new ideas for the development of evidence-based medicine.

As shown in Figure 4, the analysis of pneumatic therapeutic instrument will contribute to the construction of higher level hospital intelligent service and further improve the level of hospital intelligent service by relying on classification, recommendation, association rules, text nursing, natural language processing, and other nursing methods after cesarean section. Reasonable analysis and nursing of pressure therapeutic apparatus can greatly promote the medical staff's cognition of clinical practice, optimize the diagnosis and treatment business process, formulate personalized clinical decisions in line with the characteristics of patients, improve the quality and level of medical service, and lay the foundation for the development of precision medicine.

As shown in Figure 5, massive medical big data means opportunities and challenges coexist. The air pressure therapeutic instrument integrates data of multidepartment, multitype, and multiproject and has many data features. There are many kinds of data types in the air pressure therapeutic apparatus, including structured data (such as body temperature, blood pressure, pulse, and test results), semistructured data (such as medical history information, course record, and discharge summary), and unstructured data.

As shown in Figure 6, with the construction of the medical information platform, more and more medical processes rely on the hospital information system, which promotes the integration of the medical platform and the interconnection of medical equipment and provides convenient services for patients. At the same time, the massive data generated by the appointment, nursing, treatment, and other activities will be recorded, and the pneumatic therapeutic instrument can avoid the occurrence of 60% lower extremity venous thrombosis. The data of air pressure therapeutic instrument is dynamic, and its performance is mainly reflected in the recording of dynamic index data, such as ECG.

As shown in Table 2, the air pressure therapeutic instrument also records the diagnosis and treatment process and disease progress of patients and also has time characteristics; there are many missing values or abnormal values in the data of the air pressure therapeutic instrument, and the recording process may have errors or missing due to the different understanding of medical personnel. The data privacy of air pressure therapeutic instrument is relatively high, patients will leave a variety of medical and health data in the process of medical treatment, involving patient privacy, and data leakage may bring many troubles to patients. The data characteristics of the air pressure therapeutic instrument also bring difficulties and challenges to the nursing of the air pressure therapeutic instrument after cesarean section. How to better understand the nursing knowledge from a large number of data and put it into practice needs to be explored and studied. Based on the existing research, this part combs the analysis process of pressure therapeutic instrument based on the nursing after cesarean section and expounds the multidimensional medical knowledge management based on knowledge map according to the analysis of nursing results.

As shown in Figure 7, through the theoretical method of nursing after cesarean section, the data of the pressure therapeutic instrument is processed, and the knowledge is nursed and presented. The analysis and nursing of air pressure therapeutic apparatus cannot be separated from the practical needs, so solving the practical problems has become an important goal of the analysis and nursing of air pressure therapeutic apparatus. Based on the related problems existing in medical practice, through further analysis and refinement, scientific research problems are formed, and experiments are designed according to the concerned scientific problems.

As shown in Figure 8, medical knowledge is organized in the form of knowledge map, and a multidimensional medical knowledge base management system is constructed to realize multidimensional medical knowledge management. It mainly includes the construction of medical knowledge map, the design and implementation of knowledge base management system, and knowledge application. Through the knowledge discovery of pneumatic therapy instrument, we can build medical knowledge system, provide support for clinical decision-making, and solve the problem of doctors' knowledge limitations. Knowledge mapping transforms things in the real world, and the relationship between things into entities in knowledge mapping and the relationship between entities to describe knowledge is also a key problem.

On the one hand, it can promote the generation of air pressure therapeutic apparatus; on the other hand, it can enable practice. As shown in Figure 9, the intelligent generation of air pressure therapeutic apparatus, the current air pressure therapeutic apparatus also largely depends on the doctor's input, and its writing occupies a lot of time in the doctor's daily work. According to statistics, doctors spend about 6-11 hours on the air pressure therapeutic instrument documents on weekdays, which makes doctors devote a lot of energy to the writing of the air pressure therapeutic instrument, reduces the effective time for doctors to serve patients, and largely restricts the service ability of medical personnel who are already relatively scarce.

The intelligent writing of pneumatic therapeutic instrument will provide ideas for reducing the writing pressure of pneumatic therapeutic instrument. The intelligent writing of pneumatic therapeutic instrument will further improve the generation efficiency of pneumatic therapeutic instrument, reduce the writing task of pneumatic therapeutic instrument, and also help to improve the service ability and level of medical staff. The intelligent generation of air pressure therapeutic instrument based on the nursing after cesarean section includes important parts such as the cocreation of air pressure therapeutic instrument between doctors and patients, personalized template recommendation of air pressure therapeutic instrument, and structured data reasoning generation. The results of intelligent generation of air pressure therapeutic instrument are shown in Table 3.

As shown in Figure 10, in the process of intelligent generation of barometric therapeutic apparatus, patients can be guided to participate in the generation of their own barometric therapeutic apparatus by relying on the interactive characteristics of the Internet, and some information collection can be moved to the front end of patients, so as to realize the co creation of doctors and patients and reduce the editing pressure of medical personnel on barometric therapeutic apparatus. As an important information standard of air pressure therapeutic instrument, the template of air pressure therapeutic instrument determines the style and basic structure of air pressure therapeutic instrument, which can promote the standardization and integrity of medical data record. Different diseases have special requirements for the template of pneumatic therapeutic instrument, and the selection of a large number of standardized templates and the combination of each module is also a choice for medical personnel.

### 4.2. Discussion

Based on the nursing after cesarean section, according to the actual needs of patients, disease types, and conditions, the personalized template of pneumatic therapeutic instrument is automatically recommended, which will further improve the generation efficiency of pneumatic therapeutic instrument. In addition to structured data display, there are also unstructured data such as doctor's care and summary, such as admission care and discharge summary; unstructured data reasoning generation is also an important way for the intelligent survival of the air pressure treatment instrument. Some related researches have discussed the automatic generation method of Chinese discharge summary. Based on the doctor's thinking logic, nonstructured data such as nursing and abstract can be generated according to the referential data information. The doctor can further improve the generated content. The combination of human and computer will further improve the generation efficiency and quality of the pneumatic therapeutic instrument.

Decision support based on multidimensional medical knowledge system of the current medical knowledge system mainly comes from the expert knowledge of expert doctors (including explicit knowledge such as research literature and tacit expert knowledge). With the accumulation of medical health data and the development of nursing technology after cesarean section, mode discovery based on nursing after cesarean section has gradually become an important source of medical knowledge system. Together with expert knowledge, it forms a multidimensional medical knowledge system to provide support for medical decision-making. Based on the characteristics of “Internet plus medical health,” combining with the theories of cesarean section nursing, evidence-based medicine, doctor-patient codecision-making, knowledge management, and decision science, this paper constructs a multidimensional medical knowledge system decision-making framework. As an important method to support clinical decision-making, the analysis of pressure therapeutic apparatus based on the nursing after cesarean section will have an important impact on the rating of pressure therapeutic apparatus in hospital.

## 5. Conclusions

In clinical practice, disease nursing largely depends on doctors' professional ability and experience and knowledge. For doctors who lack professional ability or experience and knowledge, disease nursing has certain subjectivity, which may lead to the tension of medical supply side and the aggravation of doctor-patient contradiction. The air pressure therapeutic apparatus contains a lot of knowledge, which provides great potential for auxiliary nursing. The air pressure therapeutic apparatus analyzes the medical knowledge of nursing experts and doctors, simulates doctors' nursing reasoning, and obtains more reliable nursing prediction. The analysis and nursing of air pressure therapeutic instrument can enable disease prediction and assessment. Based on the demographic, symptoms, clinical, examination, and other related information of patients, the prediction of possible diseases and the evaluation of the severity of the disease can provide support and reference for the relevant nursing of medical staff and also has important significance for the follow-up treatment measures. Based on the support of multidimensional medical knowledge system, with the help of doctor's experience and patient's knowledge, doctors and patients make joint decisions and adopt the clinical diagnosis and treatment mode, nursing mode, and rehabilitation mode suitable for patients. The accumulated diagnosis and treatment data will also supplement and update the existing data, so as to further improve the medical knowledge system and form a treatment management cycle.

## Figures and Tables

**Figure 1:** Obtain real-time air pressure information of the patient.

**Figure 2:** Theoretical methods of nursing after cesarean section.

**Figure 3:** RCT clinical decision.

**Figure 4:** Hospital smart service construction.

**Figure 5:** Massive medical big data.

**Figure 6:** Construction and deepening of medical information platform.

**Figure 7:** Theoretical methods of postoperative care.

**Figure 8:** Organize medical knowledge in the form of knowledge graph.

**Figure 9:** The nursing process after cesarean section.

**Figure 10:** Intelligent generation process of air pressure therapy instrument.

**Table 1:** Analysis and utilization framework of air pressure therapy instrument.

Item	Collection	Extract	Storage	Capacity	RCT	Construction
Relying on classification	1.06	2.08	4.76	4.73	3.02	5.75
Recommend	0.6	3.71	2.41	1.18	3.42	2.02
Association rules	2	2.05	2.14	1.9	4.47	3.35
Text mining	0.19	3.99	2.73	1.63	4.7	6.02
High fidelity number	1.92	2.4	3.41	2.79	4.36	2.79

**Table 2:** Air pressure therapy device and record of disease progression.

Item	Data storage	Disease care	Collection	Extract	Storage	Processing capacity
Construction	1.19	1.47	1.95	3.3	3.91	1.23
Classification	5.23	2.36	4.07	3.82	3.85	4.27
Recommend	4.97	5.05	1.17	2.16	4.11	5.29
Association	4.53	3.68	1.36	2.88	2.9	3.44
Text mining	3.4	4.93	6.8	2.18	1.49	4.43

**Table 3:** The result of intelligent generation of air pressure therapy instrument.

Item	Collection	Extract	Storage	Demand M	Data storage	Disease care
RCT	2.51	1.19	1.47	1.95	3.3	3.91
Construction	5.22	5.23	2.36	4.07	3.82	3.85
Classification	1.2	4.97	5.05	1.17	2.16	4.11
Recommend	1.57	4.53	3.68	1.36	2.88	2.9
Association	1.73	3.4	4.93	6.8	2.18	1.49

## Data Availability

No data were used to support this study.
